# Seroprevalence of Anti-tTg-IgA among Symptomized Celiac Disease Patients and Their Correlation with Rotavirus Infection

**DOI:** 10.1155/2022/6972624

**Published:** 2022-09-22

**Authors:** Asma Sadiq, Jadoon Khan, Irfan Ullah, Nosheen Basharat, Sajid Ali, Ahmad Ud Din, Ijaz Ali, Arshad Farid, Muddaser Shah, Mohamed M. Abdel-Daim, Ghadeer M. Albadrani, Imtiaz Ali Khan

**Affiliations:** ^1^Department of Microbiology, University of Jhang, Jhang, Pakistan; ^2^Department of Microbiology, Quaid-i-Azam University, Islamabad, Pakistan; ^3^Department of Life Sciences, School of Science, University of Management and Technology (UMT), Lahore, Pakistan; ^4^Molecular Virology Laboratory, Department of Biosciences, COMSATS University, Islamabad, Pakistan; ^5^Institute of Biotechnology and Microbiology, Bacha Khan University, Charsadda, Pakistan; ^6^Institutes for Systems Genetics, West-China Hospital, Sichuan University, China; ^7^Gomal Center of Biochemistry and Biotechnology, Gomal University, D.I. Khan 29059, Pakistan; ^8^Department of Botany, Abdul Wali Khan University Mardan, Mardan 23200, Pakistan; ^9^Natural and Medical Sciences Research center, University of Nizwa, P.O. Box 33, Birkat Al Mauz, Nizwa 616, Oman; ^10^Department of Pharmaceutical Sciences, Pharmacy Program, Batterjee Medical College, P.O. Box 6231, Jeddah 21442, Saudi Arabia; ^11^Pharmacology Department, Faculty of Veterinary Medicine, Suez Canal University, Ismailia 41522, Egypt; ^12^Department of Biology, College of Science, Princess Nourah bint Abdulrahman University, P.O. Box 84428, Riyadh 11671, Saudi Arabia; ^13^COMSATS University, Islamabad, Abbottabad Campus, Abbottabad, KP, Pakistan

## Abstract

Celiac disease (CD) is a chronic inflammatory disorder in the intestinal tract as a response to the use of gluten in genetically predisposed individuals. It is a worldwide problem, with a high prevalence rate in North America. This is a descriptive cross-sectional study involving 1090 samples collected from different hospitals of Rawalpindi and Islamabad, Pakistan, from January 2019 to December 2019. In this study, 1090 blood samples screened for seroprevalence of anti-tTG antibodies in CD symptomatic patients via ELISA (enzyme-linked immunosorbent assay). 1090 fecal samples from the same CD patients were collected and tested for the presence of rotavirus (RV) via ELISA and RT-PCR. Of the 1090 patients tested for seroprevalence of anti-tTG antibodies, 112/1090 (10.3%) were found to be positive. Of the 112 anti-tTG-positive patients, 78/112 (70%) were positive for RV via ELISA and 74/112 (66.1%) were RV positive via RT-PCR. A statistically significant association was reported between rotavirus infection and celiac disease (*p*˂0.05). Anti-tTG antibodies were higher in age group 6 (12-18 years) patients (18.4%) and at minimum in age group 3 (1-3 years) patients (4.8%). However, there was a statistically insignificant relationship between group age and CD prevalence (*p* > 0.05). The highest CD prevalence was noted during winter season (19.6%) and the lowest (3.0%) during fall/autumn. Our study findings demonstrate that Pakistan has a high prevalence of CD compared to other studies. Further studies in the fields of environmental risk factors and treatment with more advanced serological and histopathological studies are needed in the future.

## 1. Introduction

Celiac disease (CD) is a chronic disorder marked by an abnormal immune response in genetically susceptible people triggered by gluten proteins present in wheat, rye, and barley, as well with HLA-DQ2/DQ8 acting as a biological risk factor [1–3]. Previously, this disease was known to be more common to the American population, but prevalence studies have shown that CD is a globally widespread disease [4]. According to recent estimates, 1% of the world's population has celiac disease [5]. Currently, 90% of people with CD contain the human leukocyte antigen DQ2 haplotype, while the remaining 10% have the DQ8 haplotype. DQ2 is present in the white population of western Europe, northern and western Africa, the Middle East, and central Asia, while DQ8 is widespread in people from Latin America and northern Europe [6].

Celiac disease was first identified by Samuel Gee in 1888, and the role of gluten in the root of its pathology became clearer in 1953 [7]. Gluten is the common term for alcohol-soluble proteins found in different cereals, particularly wheat, spelt, kamut, rye, and barley [8]. Generally, gluten proteins are enriched in glutamine and proline residues [9]. Their high proline content renders them vulnerable to hydrolysis induced by human gastrointestinal tract proteases [10]. Several hypotheses have proposed that the globalization and widespread distribution of “fake” or “extreme” versions of the Mediterranean diet, including the ingestion of very large amounts of gluten (up to 20 g/day), has led to an increased prevalence rate of CD [11]. Moreover, gluten quality itself may also serve as a contributing factor. Consequently, the development of new grain varieties may have affected the increased number of CD cases recently [12]. These observations have not, however, been verified, and the real cause of the risk remained unclear in CD diagnoses.

The epidemiological finding that similar “outbreaks” are identified in the Western world for other autoimmune diseases indicates that there may be environmental factors other than gluten at play [13]. The main “environmental factors” such as the type and pattern of milk-feeding and breast-feeding may also play a role, affecting the intestinal microenvironment [14]. In celiac cases, the intake of gluten causes enteropathy with compromised mucosal surface and, ultimately, malabsorption and diarrhea [15]. If treatment is delayed, CD may cause complications related to iron deficiency, fertility problems, bone fracture, alopecia, extraintestinal autoimmune abnormalities, and cancer [16–18].

Patients having celiac disease have a higher risk of concomitant autoimmune disorders (5%), while patients with autoimmune diseases, mainly those with diabetes or thyroid disease, sometimes develop celiac disease [19]. It has been reported that there is a connection between CD and several rheumatic disorders. Juvenile idiopathic arthritis (JIA) is known as chronic arthritis with an autoimmune aetiology, and CD is connected with susceptibility to JIA [20]. CD prevalence has also been observed to be higher in persons with autoimmune liver disorders [21]. The occurrence of autoimmune thyroiditis (AT) in celiac disease (CD) is well documented in adults but less so in children [22].

The European Society for Pediatric Gastroenterology, Hepatology and Nutrition (ESPGHAN) has proposed criteria for the diagnosis for CDs. The recommendations are based on gluten-dependent signs, CD-specific antibodies levels, HLA-DQ2 and/or HLA-DQ8, and histopathological observations, villous atrophy, and crypt hyperplasia, in a duodenum biopsy [23].

There are many other indications that involve infectious agents, especially viruses that trigger CD [24]. Infections with adenovirus, enterovirus, hepatitis C virus, and rotavirus are correlated with greater CD incidence [25, 26]. Wild-type rotavirus (RV) infection has been reported as a possible risk factor for CD development [27]. In severe celiac disease, the viral protein VP7 is recognized by a subset of antitransglutaminase IgA antibodies, indicating a potential role of rotavirus infection in disease pathogenesis via a molecular mimicry process [28, 29]. Two studies identified the possible protective effect of oral attenuated RV vaccination in reducing CD incidence in vaccinated children [29, 30]. However, despite the empirical and clinical ramifications of pathogenic organisms serving as CD causes, nothing is understood about the mechanisms through which the disease is triggered by infectious agents.

As many of the aspects of the celiac disease is unclear however according to the facilities and requirement available in Pakistan, the current study is designed to evaluate the presence of anti-tTg-IgA antibodies among the celiac disease symptomized patients and frequency of rotavirus among them through serological and molecular analyses.

## 2. Material and Methods

### 2.1. Ethical Approval

The ethical approval of the study was taken from Sarhad University ethical review committee and Pakistan Institute of Medical Sciences (PIMS) Hospital, Islamabad, Pakistan.

### 2.2. Study Design

A descriptive cross-sectional study was designed in Pakistan's capital-territorial hospitals between 1 January 2019 and 31 December 2019 to investigate the seroprevalence of anti-tTg-IgA antibodies in patients with symptoms of celiac disease and their correlation with rotavirus infection.

### 2.3. Sample Collection

A total of 1090 patients were studied at different hospitals of the capital territory of Pakistan. The list and number of samples taken from each hospital are given in Table 1. Following the medical officer's observation of symptoms, an informed written questionnaire including age, gender, family history of celiac disease, and 5 cc of venous blood samples and stool samples were obtained from each patient. The samples were aseptically transferred to the molecular virology laboratory of COMSATS University, Islamabad, for serological and molecular characterizations of the disease.

### 2.4. Inclusive and Exclusive Criteria

The patients from different age groups and genders, suspected of having celiac disease on the basis of medical symptoms, and having no genetic, diabetic, and already previous celiac disease history were included in the study. Those patients which are already positive for celiac disease and diabetic or any other hereditary/genetic disease were excluded from the study.

## 3. Serological Assays

### 3.1. Detection of IgA Antitissue Transglutaminase (tTG) Antibodies via ELISA

Following centrifugation of blood samples, the serum was isolated, and titer of IgA antitissue transglutaminase (tTG) antibodies was determined using the enzyme-linked immunosorbent assay (ELISA) with the help of the human tTG recombinant antigen (Genesis Diagnostics, Cambridgeshire, UK). The human serum samples were diluted with water (1 : 100) followed by incubation at room temperature for half an hour and then washed for three times. The horseradish peroxidase-labeled rabbit antihuman IgA were mixed and subsequently incubated at room temperature for 30 minutes. Optical density (OD) was read at 450 nm. According to the standard procedure, the results were noted in arbitrary units (AU). According to the manufacturer instruction of the kit, the cutoff value of 7 AU was considered as positive.

### 3.2. RVA Detection by Enzyme Immunoassay (ELISA)

Fecal dilutions (10%) were prepared and tested for the detection of RVA antigen by using ProSpectT ELISA Rotavirus Kit (Oxoid Ltd., UK).

### 3.3. Nucleic Acid Extraction

Fecal dilutions (10%) were freshly prepared for RNA extraction. The extraction of the RNA was carried out using the QIAamp viral RNA minikit (Qiagen, The Netherlands) in compliance with the company's instructions.

### 3.4. Molecular Analysis of VP4 and VP7 Genes through RT-PCR

RT-PCR was performed for two RVA outer capsid proteins (VP7, 1062 bp, and VP4, 876 bp). Consensus primers used in the current study are previously described by Sadiq et al. [31]. The RNA template was subjected to denaturation for 2 minutes at 95°C. The reverse transcriptase PCR (RT-PCR) was then performed by using the commercially available Qiagen OneStep RT-PCR Kit (Qiagen, The Netherlands). The RT-PCR parameters are used as described by Sadiq and her colleagues [32] and included initial reverse transcription (at 50 C for 30 min), polymerase activation (at 95°C for 15 min), 40 cycles of amplification (denaturation: at 94°C for 45 s), annealing for VP4 (at 45°C for 45 s) and annealing for VP7 (at 50°C for 45 s), product extension (at 72°C for 1 min), and final extension (at 72°C for 10 min). After completion of RT-PCR, the resulting PCR products were subjected to polyacrylamide gel electrophoresis, further stained with ethidium bromide (EtBr, Sigma Aldrich), and envisioned on ultraviolet light (UV-light).

### 3.5. Statistical Analysis

Statistical analyses were conducted through Statistical Package for Social Science (SPSS version 16.00). Regression analysis was carried out for the seroprevalence of celiac disease between different individuals and the correlation with rotavirus; the data are shown in the tables keeping significance where *p* < 0.05.

## 4. Results

### 4.1. Celiac Disease Seroprevalence and Sociodemographic Characteristics

A total of 1090 patients were studied for seroprevalence of anti-tTg IgA, and 112/1090 (10.3%) were found to be seropositive. Of the 1090 samples, 678 were female and 412 were male. There was a statistically insignificant correlation for the gender-wise distribution of celiac disease (*p* > 0.05) as shown in Table 2. The total patients were divided into 6 age groups as shown in Table 2. Anti-tTg-IgA antibodies were higher in age group 6 (12-18years) patients (18.4%) followed by age group 5 (6-12 years) patients (15.2%), age group 4 (3-6 years) patients (12.8%), age group 2 (1 month to 1 year) patients (7.9%), and age group 1 (0 days to 10 months) patients (7.1%) and at minimum in age group 3 (1-3 years) patients (4.8%), but the age group was also found to be statistically nonsignificant (*p* > 0.05) as shown in Table 3.

### 4.2. Season-Wise Distribution of Celiac Disease

According to the timeframe of the study, the patients were studied in four seasons of the year while the highest prevalence was noted during winter season (19.6%) followed by spring (12.4%) and summer (10.9%) while the lowest flow (3.0%) was observed during fall/autumn as shown in Table 4. There is statistically insignificant association between seasonality and CD prevalence (*p* > 0.05).

### 4.3. Molecular Analysis of Rotavirus among Anti-tTg-IgA-Positive Individuals

RVA was detected through ELISA in 78 out of 112 celiac-positive samples. The ELISA-positive samples were subjected to molecular analysis (RT-PCR). The molecular analysis of rotavirus among anti-tTG IgA-positive individuals confirmed that 74/112 (66.1%) of individuals positive for anti-tTg- IgA antibodies were infected with rotavirus also. Statistically significant association was observed between celiac disease and rotavirus infection (*p* < 0.05) (Table 5).

## 5. Discussion

Celiac disease (CD) is a complex disorder arising from the combination of genetic and environmental factors [33]. Owing to several factors, the epidemiological picture of CD in the world is changing, e.g., more knowledge of the large variance in the clinical manifestations of CD and the discovery of new serological markers that are easier and cheaper and contribute to an improvement in the detection ability and thus an increase in the estimated prevalence of CD [34, 35].

In this descriptive cross-sectional study, seroprevalence of anti-tTG-IgA antibodies in blood samples of patients suspected of CD was determined via ELISA. In addition, fecal samples from the same patients were also tested for RVA infection via ELISA and RT-PCR. The seroprevalence for anti-tTG-IgA antibodies detected in CD patients is 10.3% (112/1090). Similar prevalence studies have been performed in other countries around the world. A study conducted in Colombia in 2020 has reported overall seroprevalence for anti-tTG of 4.82% [36]. In two Brazilian studies performed on blood bank donors, they find a seroprevalence of 0.28-0.60% [37, 38]. In Mexico, Argentina, and Brazil, the largest epidemiological studies have been conducted, with a discrepancy between reported CD prevalence and seroprevalence ranging from 0 to 3.03% [37, 39–43]. In a study performed in Iran in 2008, a prevalence rate of 0.5% was reported [44]. However, another study performed in Turkey showed a comparable prevalence of 8.3% in patients with risk factors, such as dwarfism, using intestinal endoscopic biopsy [45]. Similar results have also been reported in a Pakistani study with a seroprevalence for anti-tTG-IgA antibodies of 11.7% [46]. The low seroprevalence of celiac disease in countries relative to our study may be attributed to their high sample size or false-negative ELISA findings. Similarly, high seroprevalence could be due to large sample size and false-positive ELISA results.

Recently, it has been reported that CD more frequently occur in females, and in the adult population, there is a growing incidence of the disease with age [47]. In the present study, the prevalence of CD is high in females than in males. Similar findings for high female prevalence are also documented in other world studies [48]. A similar study from Pakistan revealed high female prevalence rate (60%) than male (40%) [49]. A study of 21 subjects found that the majority of patients with celiac disease were women (male/female 1 : 2.5) [50]. A study in the United Arab Emirates (UAE) showed higher CD prevalence in women (1 : 44) [51]. In Pakistan, a study found that male gender was mainly affected compared to females [46].

The quantity of gluten intake and the degree of intestinal damage are unknown factors that lead to the increased prevalence of latent CD amongst women [51]. There are reports that autoimmune disorders have common genetic risk factors, many of which are gender-based [52]. Women are likely to be genetically more vulnerable to environmental factors that influence the immunological patterns leading to the development of CD. A study reported that smoking could be CD-protective because some CD patients who were smokers had negative CD serology confirmed by endoscopy [53] which is supported by further studies [52, 54]. Gliadin, an ingredient of wheat gluten considered to be a significant factor in the aetiology of celiac disease, is associated with many other diseases by increasing its effect on intracellular intestinal motility [55]. Since the activation of T cells in the gastric mucosa by gliadin is a key initiative in the progression of the mucosal inflammation of celiac disease, smoking can alter the ability of T cells to respond to gliadin and thus reduce the risk of developing celiac disease [56]. According to a survey conducted in Pakistan in 2012, the estimated prevalence rate of smoking was 15.2% overall, 26.6% among males and 0.4% among females [57]. Smoking can also partly explain why the prevalence of celiac disease in males was much lower in this study compared to females. On the other side, the gender difference could be due to the inability of the immunological test to check the disorder in young men due to hormonal or environmental changes. It is suggested that even in young men with clinical manifestations indicative of the disorder, endoscopy and biopsy ought to be the criteria for diagnosis with very little focus on serological tests [51].

CDs significantly affect people of all ages and all races around the world. Two CD peaks are visible: in infancy (<6-year-old) and in the 4th-5th decade. In paediatric patients, classical presentation is also documented in other world studies [48]. A similar study from Pakistan revealed high female prevalence rate (60%) than male (40%) [49]. A study of 21 subjects found that the majority of patients with celiac disease were women (male/female 1 : 2.5) [50]. A study in the United Arab Emirates (UAE) showed higher CD prevalence in women (1 : 44) [51]. In Pakistan, a study found that male gender was mainly affected compared to females [46].

CDs significantly affect people of all ages and all races around the world. Two CD peaks are visible: in infancy (<6-year-old) and in the 4th-5th decade. In paediatric patients, classical presentation is more normal and appears to occur early in life (6-24 months), while atypical presentation normally occurs later (>5-year-old) and in adults [7, 58]. In our study, the prevalence of CD is high in adolescents (12-18 years of age) (18.4%) and at minimum in newborn (0-10 months) patients (7.1%). A study from Pakistan showed similar high CD prevalence rate in adolescents (up to 14 years of age) [46]. Another Pakistani study reported a mean age of 6 years for the initiation of signs and symptoms of CD [59]. Two other studies from UAE and USA reported high CD prevalence in the age group 16-30 years [51, 60]. CD was also shown to be higher in children (1 : 71) than in adults (1 : 357) in a study conducted in Spain [50]. In the present study, the highest prevalence of CD disease is reported during winter season (19.6%) while the lowest (3.0%) in the fall/autumn season. A similar study from Pakistan has reported highest prevalence (33.4%) in spring season and lowest prevalence (15.8%) in winter season [46]. A recent research indicates that the risk of disease can be related to the seasons and place of birth. Based on user data from approximately 2 million Swedish children born between 1991 and 2009, researchers discovered that, comparative to winter babies, those delivered in spring, summer, and fall had an 8-10 percent increased risk of developing celiac disease [61]. A study in Sweden reported vitamin D deficiency could be correlated with seasonal changes in birth shown in autoimmune disorders, such as CD [61, 62].

Rotavirus is the main cause of severe gastroenteritis in infants and toddlers around the world. It is a leading cause of death in low-income countries and a significant cause of morbidity in developed countries [63]. Rotavirus infects intestinal wall and induces gastroenteritis; nevertheless, infection is not restricted to intestinal epithelium, and systemic viral spread has also been frequently documented [64]. We have investigated in the current study the correlation between CD and RV infection. A total of 1090 fecal samples from all of those patients were collected from which blood samples were taken for CD serological analysis and tested for RVA via ELISA and RT-PCR. Of the 112 anti-tTG IgA-positive patients, 74/112 (66.1%) were also infected with RV. A related research in Iran reported the identification of the rotavirus VP6 gene in 8/25 (32%) patients with positive CD serology [65]. In a prospective study, a high prevalence of rotavirus infections has been reported to increase the risk of autoimmune celiac disease in childhood in genetically susceptible individuals [66]. There are some drawbacks to this study. The study included patients aged 0 days to 18 years. Older age groups should also be included in future research. In addition, samples should be obtained from hospitals in major cities throughout the country. The study includes only the key risk factors for CD and does not consider factors that could defend against CD, like smoking. In the identification of celiac disease, serological diagnosis is critical employing specific immunological markers, but the true prevalence is not confirmed until histopathological diagnosis.

## 6. Conclusions

In summary, this is the first study in Pakistan to lead us to believe that frequent rotavirus infections may be a cause of early childhood autoimmune celiac disease. Few researchers have investigated the role of specific gastrointestinal infections in celiac disease. We propose that tTG-IgA would be an effective marker for massive CD monitoring and that when tTG-IgA levels are too low to be detectable, some powerful complementary tests should be used. Furthermore, more advanced serological and histopathological studies are welcomed in the future that may lead to a reliable and more effective diagnosis. Future research can use tests that can take a number of patient measurements at once and can then be combined to enhance sensitivity and specificity. It is further anticipated then that an equilibrium can be found between novel tests and conventional methods to provide comprehensive insights into disease diagnosis. The findings of this study are of great significance from a health and safety point of view and should be forwarded to the public health services to raise awareness of the disease in healthcare workers and the community as a whole.

## Figures and Tables

**Table 1:** List of samples collected from the hospitals of Rawalpindi and Islamabad, Pakistan, during 2019.

Hospital	Patients studied	Percentage
Shaheen Health Plus	370	33.9%
Holy Family Hospital Rawalpindi	210	19.2%
Benazir Bhutto Hospital Rawalpindi	190	17.4%
Pakistan Institute of Medical Sciences Hospital, Islamabad	210	19.2%
District Headquarter Hospital Rawalpindi	110	10.1%
Total	1090	100%

**Table 2:** Evaluation of anti-tTG-IgA antibodies among male and females.

Celiac disease	Gender		*t*-value	*p* value	95% confidence interval		*R*-squared
	Male	Female			Lower Boundary	Upper Boundary	
Positive	68/678 (10%)	44/412 (10.6%)	-.342	0.732	-.044	.031	0.000
Negative	610/678	368/412					
Total prevalence	112/1090 (10.3%)						

**Table 3:** Seroprevalence of anti-tTg-IgA antibodies among different age group patients.

Age groups	(Months/years)	Celiac disease	*t*-value	*p* value	95% confidence interval		*R*-squared
		Infected/total (%)			Lower Boundary	Upper Boundary	
Age group 1(newborn)	(0 days to 10 months)	2/28 (7.1)	-.697	0.486	-.235	.112	0.018
Age group 2 (infants)	(1 month to 1 year)	26/328 (7.9)	-.730	0.466	-.199	.091	
Age group 3 (toddler)	(1 to 3 years)	10/208 (4.8)	-1.177	0.239	-.229	.057	
Age group 4 (preschool)	(3 to 6 years)	50/390 (12.8)	-.050	0.960	-.147	.139	
Age group 5 (school age child)	(6 to 12 years)	10/66 (15.2)	.261	0.794	-.136	.177	
Age group 6 (adolescent)	(12 to 18 years)	14/76 (18.4)	.674	0.500	-.101	.208	

**Table 4:** Seasonal-wise distribution of anti-tTg-IgA antibodies among celiac disease patients.

Characteristics	Celiac disease	*t*-value	*p* value	95% confidence interval		*R*-squared
	Infected/total (%)			Lower Boundary	Upper Boundary	
Spring	42/340 (12.4)	.082	0.935	-.060	.065	0.024
Summer	42/384 (10.9)	-.516	0.606	-.053	.031	
Fall/autumn	08/264 (3.0)	-2.758	0.006	-.155	-.026	
Winter	20/102 (19.6)	1.865	0.063	-.004	.154	

*p* < 0.05 was considered statistically significant.

**Table 5:** Rotavirus correlation among patients with celiac disease.

Celiac disease	Rotavirus		*t*-value	*p* value	95% confidence interval		*R*-squared
	Negative	Positive			Lower Boundary	Upper Boundary	
Negative	978	0	43.601	0.000^∗^	.919	1.006	0.636
Positive	112	74 (66.1%)					

*p* < 0.05 was considered statistically significant, *p* value = 0.000 is highly significant.

## Data Availability

All relevant data are available in the manuscript.
